The article "MATN1‐AS1 promotes glioma progression by functioning as ceRNA of miR‐200b/c/429 to regulate CHD1 expression" was retracted in 2024. Reasons: errors in the images; plagiarized images; overlap with other authors' work; unreliable results or conclusions.

# MATN1‐AS1 promotes glioma progression by functioning as ceRNA of miR‐200b/c/429 to regulate CHD1 expression

**DOI:** 10.1111/cpr.12700

**Published:** 2019-10-30

**Authors:** Jun Zhu, WeiTing Gu, Cai Yu

**Affiliations:** ^1^ Department of Neurosurgery Rui Jin Hospital Shanghai Jiao Tong University School of Medicine Shanghai China; ^2^ Department of Neurosurgery Rui Jin Hospital North Shanghai Jiao Tong University School of Medicine Shanghai China

**Keywords:** cell proliferation, CHD1, glioma, MATN1‐AS1, miR‐200b/c/429

## Abstract

**Objectives:**

Long non‐coding RNA (lncRNA) MATN1‐AS1 is a newfound lncRNA that has been rarely explored in cancers. Herein, we would like to investigate its role in glioma.

**Materials and methods:**

qRT‐PCR was conducted to examine gene expression in glioma. Then, MTT assay, colony formation assay and flow cytometry analysis were applied to evaluate the function of MATN1‐AS1 on glioma cells. Western blot was performed to measure the protein levels of genes. Besides, the luciferase reporter assay, RNA pull‐down assay, RIP assay and Spearman's correlation analysis were also performed as needed.

**Results:**

Firstly, a data from TCGA showed that MATN1‐AS1 might be largely implicated in glioma. Meanwhile, MATN1‐AS1 upregulation confirmed in glioma predicted poor clinical outcomes. Functionally, MATN1‐AS1 knockdown restrained cell proliferation but stimulated apoptosis in vitro and repressed tumour growth in vivo. Mechanistic investigations validated that MATN1‐AS1 functioned as a ceRNA for miR‐200b/c/429 to upregulate CHD1 which was also verified to exert a growth‐promoting role in glioma cells here. Importantly, both CHD1 overexpression and miR‐200b/c/429 inhibition could rescue the obstructive role of MATN1‐AS1 silence in glioma cells.

**Conclusions:**

MATN1‐AS1 promotes glioma progression through regulating miR‐200b/c/429‐CHD1 axis, suggesting MATN1‐AS1 as a probable target for glioma treatment.

## 1 INTRODUCTION

Glioma, one of the most prevalent and aggressive cancers attacking the central nervous system, accounts for approximately 80% of primary brain malignancies.^1^, ^2^ Glioma contains four histological subtypes, such as astrocytoma, oligodendroglioma, ependymoma and mixed tumours.^3^ Though some progresses in early diagnosis and treatment, majority of the patients with glioma are still detected at advanced stages, and clinical outcomes of them are still disappointing after treatment.^4^ Despite intensive study has been carried out for the exploration of molecules implicated in glioma cell proliferation and invasion,^5^ only limited molecular mechanisms have been uncovered and applied to the clinic so far. Therefore, studies for the discovery of novel therapeutic targets in glioma are urgently prompted.

The article "MATN1‐AS1 promotes glioma progression by functioning as ceRNA of miR‐200b/c/429 to regulate CHD1 expression" was retracted in 2024. Reasons: errors in the images; plagiarized images; overlap with other authors' work; unreliable results or conclusions.

Long non‐coding RNAs (lncRNAs), with more than 200 nucleotides in length, are a class of transcripts that cannot encode protein.^6^ Increasing evidence has shown that lncRNAs play significant roles in various biological processes including tumorigenesis in a wide range of cancers containing glioma.^7^, ^8^ For instance, the SNHG5/miR‐32 axis regulates gastric cancer cell proliferation and migration by targeting KLF4.^9^ Long non‐coding RNA HOXA‐AS2 regulates malignant glioma behaviours via the MiR‐373/EGFR axis.^10^ CRNDE promotes malignant progression of glioma by attenuating miR‐384/PIWIL4/STAT3 axis.^11^ MATN1 antisense RNA 1(MATN1‐AS1), a newfound lncRNA that locates in 1p35.2, has been recognized to be non‐significantly downregulated in ischaemic stroke.^12^ However, the function of MATN1‐AS1 needs to be discovered.

Competing endogenous RNAs (ceRNAs), which also celebrated as miRNA “sponges” or miRNA “decoy” that firstly identified in plants and named “target mimicry” process,^13^ are a class of RNA transcripts that competitively binding to the common miRNA via the base complementary with miRNA response elements (MREs), thereby reducing the amount of miRNAs targeting messenger RNAs (mRNAs).^14^, ^15^, ^16^ Recently, many lncRNAs have been found to function in cancers through such mechanism. For example, lncRNA SPRY4‐IT1 sponges miR‐101‐3p to promote proliferation and metastasis of bladder cancer cells through upregulating EZH2.^17^ Long non‐coding RNA UICLM promotes colorectal cancer liver metastasis by acting as a ceRNA for microRNA‐215 to regulate ZEB2 expression.^18^ Nevertheless, it remains covered whether MATN1‐AS1 could also implicate in a ceRNA network in glioma.

In this study, we first discover that MATN1‐AS1 may play a significant role in glioma after analysing TCGA database. Then, potential miRNAs that might have interactions with MATN1‐AS1 are screened using online tools starBase 2.0, and miR‐200b/c/429 from miR‐200 family is found out. Based on this, we aim to investigate the role and function of MATN1‐AS1 in glioma and identify whether it affects glioma by functioning as ceRNA for miR‐200b/c/429.

## 2 MATERIALS AND METHODS

### 2.1 Clinical samples

Clinical samples (n = 80) were collected from patients with glioma who underwent operations in the Rui Jin Hospital, Shanghai Jiao Tong University School of Medicine, Shanghai Jiao Tong University School of Medicine. All of these patients suffered no any treatment before surgery. The clinicopathologic features of each patient were also collected in Table 1. The using of human tissues in this study was approved by the Ethics Committee of the Rui Jin Hospital, Shanghai Jiao Tong University School of Medicine, and the informed consent had been signed by all of the patients before our study.

The article "MATN1‐AS1 promotes glioma progression by functioning as ceRNA of miR‐200b/c/429 to regulate CHD1 expression" was retracted in 2024. Reasons: errors in the images; plagiarized images; overlap with other authors' work; unreliable results or conclusions.

**Table 1:** Correlation between MATN1‐AS1 Expression and Clinical Features. (n = 80)

Variables	MATN1‐AS1 expression		χ^2^‐value	*P*‐value
	Low	High		
Age				
≤50	26	43	2.637	.185
>50	7	4		
Gender				
Male	31	38	2.800	.113
Female	2	9		
Tumour size				
<5	25	19	9.779	.003**
≥5	8	28		
KPS				
≥70	25	17	12.184	.001**
<70	8	30		
WHO grade				
Ⅰ+Ⅱ	23	18	7.650	.007**
Ⅲ+Ⅳ	10	29		

Note

Low/high by the sample median. Pearson chi‐square test.

** *P* < .01 is considered statistically significant.

### 2.2 Cell lines and cell culture

Human glioma cell lines (T98G, LN229, U87 and U251) and human embryonic kidney cell line HEK‐293T were purchased from the American Type Culture Collection (ATCC, USA), while the normal human astrocytes (NHAs) were obtained from ScienCell Research Laboratories (Carlsbad, CA, USA). All of the cells were grown in DMEM (Dulbecco's modified Eagle's medium) with 10% FBS (foetal bovine serum; Gibco, USA) and maintained in a humid atmosphere with 5% CO_2_ at 37℃.

### 2.3 Cell transfection

The specific shRNAs against MATN1‐AS1 and corresponding control shRNA (sh‐NC) as well as sh‐CHD1 and its control were obtained from Santa Cruz Biotechnology Inc (Dallas, TX, USA). Similarly, pcDNA 3.1/MATN1‐AS1 and its empty vector are obtained from RiboBio, Guangzhou, Guangdong, China. Cell transfection was conducted under the use of Lipofectamine 2000 (Invitrogen) following the manufacturer's protocol. And the sequences of shRNAs used in this study were shown as below: shMATN1‐AS1#1: CCG GCC TTG TTG TAT ACA GTC ATT ACT CGA GTA ATG ACT GTA TAC AAC AAG GTT TTT TG; shMATN1‐AS1#2: CCG GGC GCT CCT GTT TAT GTA CTT ACT CGA GTA AGT ACA TAA ACA GGA GCG CTT TTT TG; shMATN1‐AS1#3: CCG GGC TCC TGT TTA TGT ACT TAC ACT CGA GTG TAA GTA CAT AAA CAG GAG CTT TTT TG; sh‐NC: CCG CCC TTT TTT GGG CCT AAA ACC CCT GGA GGA AAA ATT GTT TTC GGC GGG GTA GTC CG; sh‐CHD1: CCG GCA AGC AAG ACA GCA GAT ATT ACT CGA GTA ATA TCT GCT GTC TTG CTT GTT TTT G; and its control sh‐NC: CCC GCC TCC GGG TCT CCC CTT TAA AAA CCC CAT TTT AAA AAC CCT AAA GGG CCC CTG G.

### 2.4 RNA extraction and qRT‐PCR

Total RNAs were extracted with TRIzol reagent (Invitrogen, Grand Island, NY). Reverse transcription was performed using Superscript III transcriptase (Invitrogen, Grand Island, NY). qRT‐PCR was carried out in a Bio‐Rad CFX96 system, and SYBR Green was utilized to examine the mRNA level of genes. To normalize the expression of genes, GAPDH was used as a control in this study. All experiments were performed for at least three times.

The article "MATN1‐AS1 promotes glioma progression by functioning as ceRNA of miR‐200b/c/429 to regulate CHD1 expression" was retracted in 2024. Reasons: errors in the images; plagiarized images; overlap with other authors' work; unreliable results or conclusions.

### 2.5 Cell proliferation assay

Cells were seeded into 24‐well plates at a density of 3000 cells/well and cultured for 24, 48, 72 and 96 hours. Then, culture solution containing MTT was used to replace the medium, and DMSO was applied to melt the blue crystals. At last, cell viability was estimated by detecting the absorbance at 490 nm. All tests were carried out in triplicate.

For colony formation assay, cells with a concentration of 1 × 10^3^ cells/well were seeded into six‐well plates and cultured in DMEM supplemented with 10% FBS at 37℃. After incubated for two weeks, cells were washed using PBS and fixed with methanol followed by staining with 1% crystal violet. Thereafter, the number of colonies was counted manually. All tests were carried out in triplicate.

### 2.6 Flow cytometry analysis

After incubation for two days, the harvested cells were used for following experiments. For analysis of cell cycle, cells were fixed by 75% ethanol and then stained using PI (BD Biosciences). FACScan was applied to analyse the stained cells, and then, the proportion of cells in different cell cycle phases (G0/G1, G2/M and S) were calculated.

In cell apoptosis analysis, apoptosis rate of transfected cells was evaluated by using Annexin V‐APC/PI apoptosis detection kit (KeyGEN) following the manufacturer's instruction and then analysed using FACScan. All tests are carried out in triplicate.

### 2.7 In vivo experiment

The male nude mice at the age of 4 weeks were obtained from the Shanghai LAC Laboratory Animal Co. Ltd. (Shanghai, China). Then, each mouse was injected with U87 cells (at a density of 1 × 10^7^ cells per 100 μL) transfected with either control or sh‐MATN1‐AS1 at their left flank. Then, the tumour volume was assessed by calliper measurements every four days and calculated according to the following formula: volume = length × width^2^/2. After that, the mice were sacrificed after injection for five weeks, and the tumours derived from each mouse were excised and photographed. Subsequently, the tumours were weighed and then fixed for IHC staining. This study was carried out according to the Care and Use of Laboratory Animals of the National Institutes of Health.

### 2.8 Immunohistochemistry (IHC) staining

Paraffin sections made from tumours obtained from in vivo experiments were used for immunohistochemistry assays to detect protein expression levels of Ki67 proteins. In accordance with the manufacturer's introduction, tissue sections stained immunohistochemically are determined separately by two pathologists using the indirect streptavidin‐peroxidase method. The primary antibodies against Ki67 (#9449, Cell Signaling Technology, Danvers, MA, USA) and horseradish peroxidase‐conjugated IgG were used in this study. Then, the proteins were visualized in situ by the use of 3, 3‐diaminobenzidine kit (BioGenex, Fremont, CA, USA).

The article "MATN1‐AS1 promotes glioma progression by functioning as ceRNA of miR‐200b/c/429 to regulate CHD1 expression" was retracted in 2024. Reasons: errors in the images; plagiarized images; overlap with other authors' work; unreliable results or conclusions.

### 2.9 Luciferase reporter assay

Firstly, pmirGLO‐MATN1‐AS1‐WT or pmirGLO‐MATN1‐AS1‐mut, pmirGLO‐CHD1‐wt or pmirGLO‐CHD1‐mut was constructed using a pmirGLO Dual‐luciferase Target Expression Vector (Promega, Madison, WI, USA). And miR‐200b/c/429 mimics/inhibitors (for miR‐200b/c/429 overexpression/inhibition, respectively) or miR‐NC was also obtained from RiboBio. Thereafter, these plasmids were appropriately transfected into glioma cells or Hek‐293T cells using Lipofectamine 2000 (Invitrogen, Carlsbad, CA, USA) based on the manufacturer's guide. The relative luciferase activity was determined by a dual‐luciferase reporter assay kit (Promega) after 48 hours of transfection.

### 2.10 RNA immunoprecipitation (RIP) assay

In this study, EZMagna RIP kit (Millipore, Billerica, MA, USA) was used for RNA immunoprecipitation on the basis of manufacturer's protocol. U87 and U251 cells were scraped off from the plates and dissolved in 100% RIP lysis buffer. Then, extracted cells were kept in RIP buffer, in which magnetic bead (Millipore)‐incubated human anti‐Ago2 antibody (Millipore) was contained. And beads with IgG were used as negative control. Moreover, the density of RNA was evaluated using a NanoDrop spectrophotometer (Thermo Scientific), whereas the quality of RNA was assessed by bioanalyser (Agilent, Santa Clara, CA, USA). At length, the purified RNA was analysed by qRT‐PCR. All tests were carried out in triplicate.

### 2.11 RNA pull‐down assay

RNA pull‐down assays were conducted as previously described.^17^ Briefly, RNAs were biotin‐labelled using Biotin RNA Labeling Mix (Roche) and transcribed with T7/SP6 RN polymerase (Roche Diagnostics, Indianapolis, IN, USA). Afterwards, the biotinylated RNAs were incubated with U87 and U251 cell lysates followed by the incubation of M‐280 streptavidin magnetic beads (Invitrogen, San Diego, CA, USA). After washing with buffer, the bound RNAs were evaluated by qRT‐PCR, and the eluted proteins were examined by Western blot analysis.

### 2.12 Western blot assay

First of all, proteins were extracted from cells by using RIPA buffer with 1% PMSF and the concentration of protein is evaluated by BCA assay. And then, the proteins were segregated by SDS‐PAGE and electrophoretically transferred onto PVDF membranes (Millipore, Billerica, MA). Then, the membranes were blocked with bovine serum albumin (BSA) (Sigma‐Aldrich, St. Louis, MO) and treated with specific antibodies. GAPDH protein is the loading control. The primary antibodies were as following: Bcl‐2 (#4223), Bax (#2772), CDK4 (#12790), Cyclin D1 (#2978) (above antibodies were from Cell Signaling Technology, Inc, Danvers, MA, USA), GAPDH (ab8245, Abcam) and CHD1 (20576‐1‐AP, Protein‐Tech). The secondary antibody was Rabbit Anti‐Mouse IgG H&L (ab6728, Abcam). Next, ECL chemiluminescent detection system (Thermo Fisher Scientific, Rochester, NY) was applied to visualize protein bands. In the end, all of the proteins were exposed to X‐ray film. All experimental steps were performed for at least three times.

The article "MATN1‐AS1 promotes glioma progression by functioning as ceRNA of miR‐200b/c/429 to regulate CHD1 expression" was retracted in 2024. Reasons: errors in the images; plagiarized images; overlap with other authors' work; unreliable results or conclusions.

### 2.13 Statistical analysis

GraphPad Prism (GraphPad Software Inc) was utilized for statistical analyses. Data obtained from at least three experiments are represented as a manner of means ± SD. Student's *t* test was used to analyse the differences between two groups, and one‐way ANOVA was used for multiple comparisons. Kaplan‐Meier analysis and the log‐rank test were applied to determine survival curve. The associations between clinical parameters and prognosis were assessed by using Cox regression analysis. Correlations among MATN1‐AS1, miR‐200b/c/429 and CHD1 were determined by Spearman's correlation analysis. Data were considered to have statistical significance when *P* < .05.

## 3 RESULTS

### 3.1 MATN1‐AS1 is highly expressed in glioma tissues and cell lines

To find out lncRNAs related to glioblastoma, data from TCGA database are initially analysed, and we observed that MATN1‐AS1 level was significantly related to the outcome of patients with glioma (Figure 1A). Based on this, we hypothesized that MATN1‐AS1 might play a key role in glioma. Thereby, we tested the expression levels of MATN1‐AS1 in 80 pairs of glioma tissues and adjacent non‐tumour tissues by RT‐qPCR. The results showed that MATN1‐AS1 was markedly highly expressed in glioma tissues in comparison with corresponding non‐tumour tissues (Figure 1B). Also, MATN1‐AS1 expression in glioma cell lines (T98G, LN229, U87 and U251) and normal human astrocytes (NHAs) were detected. Consistently, MATN1‐AS1 was revealed to be obviously upregulated in glioma cell lines compared with NHAs (Figure 1C). In the light of these results, we put a preliminary hypothesis that MATN1‐AS1 might act as a carcinogenic lncRNA in glioma.

**Figure 1:** MATN1‐AS1 is highly expressed in glioma tissues and cell lines. A, Overall survival in glioma patients (n = 169) with low (n = 84) or high (n = 85) MATN1‐AS1 expression. Data are obtained by analysing TCGA database, *P* = .01535 (*P* < .05) indicated that MATN1‐AS1 level is of great importance in glioma. B, RT‐qPCR results of MATN1‐AS1 expression in glioma tissues. Tissues are collected from patients with glioma who underwent surgery. C, MATN1‐AS1 expression in glioma cell lines was detected using RT‐qPCR. Data are shown as means ± SD. D, Kaplan‐Meier analysis of the correlation between MATN1‐AS1 expression and overall survival (OS) in 80 patients with glioma. The cut‐off value (6.24) is the median value of MATN1‐AS1 expression in above patients. ^**^ *P* < .01, compared with controls

The article "MATN1‐AS1 promotes glioma progression by functioning as ceRNA of miR‐200b/c/429 to regulate CHD1 expression" was retracted in 2024. Reasons: errors in the images; plagiarized images; overlap with other authors' work; unreliable results or conclusions.

### 3.2 The clinical significance of MATN1‐AS1 in glioma

Next, the correlation between MATN1‐AS1 expression and clinicopathological features of patients with glioma was analysed (Table I). Based on the cut‐off value (6.24), patients with glioma were divided into the high (n = 47) or the low MATN1‐AS1 expression groups (n = 33). It was showed that MATN1‐AS1 expression level was apparently correlated with tumour size (*P* = .003), KPS (*P* = .001) and WHO grade (*P* = .007). However, there was no statistical significance in the association between MATN1‐AS1 expression and age, gender, or tumour size. In addition, the level of MATN1‐AS1 could serve as an independent prognostic biomarker for glioma patients, so as some clinical features such as KPS (*P* = .033) and WHO grade (*P* = .032), while others had no impact on the prognosis (Table 2). Moreover, Kaplan‐Meier analysis revealed that glioma patients with high levels of MATN1‐AS1 usually had poor overall survival in contrast to those with low MATN1‐AS1 levels (Figure 1D). These data indicated that MATN1‐AS1 may be a novel prognostic biomarker for glioma.

**Table 2:** Multivariate analysis of prognostic parameters in patients with glioblastoma by Cox regression analysis

Variables	No. of cases	HR	95% CI	*P*‐value
Age				
≤50	69	1	0.398‐3.242	.812
>50	11	1.136		
Gender				
Male	69	1	0.617‐4.776	.300
Female	11	1.717		
Tumour size				
<5	44	1	0.488‐1.859	.886
≥5	36	0.952		
KPS				
≥70	42	1	0.266‐0.944	.033
<70	38	0.501		
WHO grade				
Ⅰ+Ⅱ	41	1	1.063‐4.003	.032*
Ⅲ+Ⅳ	39	2.063		
MATN1‐AS1 Level				
Low	33	1	0.179‐0.791	.010*
High	47	0.376		

Note

Proportional hazards method analysis shows a positive, independent prognostic importance of MATN1‐AS1 expression (*P* = .010).

* *P* < .05 is considered statistically significant.

### 3.3 Knockdown of MATN1‐AS1 affects cell proliferation and apoptosis in vitro

To study the biological role of MATN1‐AS1 in glioma, MATN1‐AS1 was silenced in U251 and U87 cells by transfecting with three different shRNAs (Figure 2A). Then, MTT assay demonstrated that cell viability in either U87 or U251 cells is markedly inhibited by all of the shRNAs targeting MATN1‐AS1, among which the sh‐MATN1‐AS1#2 elicited the highest inhibitory effect (Figure 2B). According to these two results (Figure 2A,B), the sh‐MATN1‐AS1#2 was chosen for following experiments and described just as sh‐MATN1‐AS1 subsequently. Seen from Figure 2C, knockdown of MATN1‐AS1 caused a large reduction in the number of colonies in U87 and U251 cells. Additionally, the proportion of cells arrested in G0/G1 phase were increased after silencing MATN1‐AS1 in U87 and U251 cells (Figure 2D). Moreover, MATN1‐AS1 knockdown distinctly increased the rate of cell apoptosis in both of two cells (Figure 2E). At last, Western blot analysis accordantly confirmed that the expression of cell cycle‐associated proteins (CDK4 and Cyclin D1) and anti‐apoptotic Bcl‐2 were downregulated, whereas pro‐apoptotic Bax was upregulated in U87 and U251 cells under MATN1‐AS1 silence (Figure 2F). These results revealed that silencing MATN1‐AS1 repressed cell proliferation and stimulated cell apoptosis in vitro.

The article "MATN1‐AS1 promotes glioma progression by functioning as ceRNA of miR‐200b/c/429 to regulate CHD1 expression" was retracted in 2024. Reasons: errors in the images; plagiarized images; overlap with other authors' work; unreliable results or conclusions.

**Figure 2:** Knockdown of MATN1‐AS1 affects cell proliferation and apoptosis in glioma cells. A, The expression of MATN1‐AS1 was evaluated by qRT‐PCR in U87 and U251 cells after transfecting separately with three different sh‐MATN1‐AS1 and corresponding sh‐NC. B, MTT assay was performed to examine cell viability in U87 and U251 cells under different transfections. C, Colony formation assay results of cell proliferative ability in U87 and U251 cells after silencing MATN1‐AS1. D‐E, Cell cycle distribution and cell apoptosis rate in sh‐MATN1‐AS1 or sh‐NC transfected U87 and U251 cells were tested by flow cytometry analysis. F, The levels of cell cycle‐associated proteins and apoptosis‐related proteins were detected in U87 and U251 cells transfected with sh‐MATN1‐AS1 or sh‐NC by Western blot analysis. Data are obtained from at least three experiments for mean ± SD. ^*^ *P* < .05, ^**^ *P* < .01 compared with controls

### 3.4 Silenced MATN1‐AS1 suppresses tumour growth in vivo

On the basis of the previous observations in vitro, a tumorigenesis assay was conducted in nude mice to make sure whether silenced MATN1‐AS1 inhibits tumour growth in vivo. As shown in Figure 3A, the formed tumours seemed to be smaller in the mice injected with U87 cells which were transduced with sh‐MATN1‐AS1 than in those injected with the control. Besides, the average weight of the tumours originated from MATN1‐AS1 silenced U87 cells was markedly less than that of tumours originated from the sh‐NC transfected cells (Figure 3B). Additionally, depletion of MATN1‐AS1 led to a significant reduction in the tumour growth rate (Figure 3C). Furthermore, the expression of Ki67, which served as an indicator of the proliferative activity of the tumour cells, was assessed by IHC staining and suggested to be remarkably decreased under MATN1‐AS1 suppression (Figure 3D). Collectively, silencing MATN1‐AS1 suppressed tumorigenesis in vivo.

The article "MATN1‐AS1 promotes glioma progression by functioning as ceRNA of miR‐200b/c/429 to regulate CHD1 expression" was retracted in 2024. Reasons: errors in the images; plagiarized images; overlap with other authors' work; unreliable results or conclusions.

**Figure 3:** Impacts of MATN1‐AS1 on tumour growth in vivo. A, Representative images of tumours derived from the nude mice injected with sh‐MATN1‐AS1 or sh‐NC transfected U87 cells. B, Quantitative analysis of the average tumour weights. C, Tumour volumes were assessed at the specific times shown in the diagram. D, Representative images of HE and IHC staining for Ki‐67 in the tumours originated from mice with different injections. ^**^ *P* < .01

### 3.5 MATN1‐AS1 directly targets miR‐200b/c/429 in glioma cells

Since many lncRNAs have been reported to function as ceRNAs in various cancers,^19^ we supposed that MATN1‐AS1 may also acted as a ceRNA in glioma. First of all, the cellular location of MATN1‐AS1 was measured and assessed by subcellular fractionation assay and FISH assay. It was found that MATN1‐AS1 was predominantly located in the cytoplasm of glioma cells (Figure S1A,B). Then, we seek out three miRNAs which belong to miR‐200 family that could bind with MATN1‐AS1 using online tool starBase v2.0 (http://starbase.sysu.edu.cn/browseNcRNA.php) (Figure 4A). And we constructed the wild‐type MATN1‐AS1 (MATN1‐AS1‐Wt) which contained the binding sites with miR‐200b/c/429 and mutant MATN1‐AS1 (MATN1‐AS1‐Mut) without binding sites (Figure 4B). Then, the luciferase reporter assay indicated that only the luciferase activity of MATN1‐AS1‐WT but not that of MATN1‐AS1‐Mut is cut down by miR‐200b/c/429 mimics in either U87 or U251 cells (Figure 4C). Besides, we revealed that both MATN1‐AS1 and miR‐200b/c/429 were apt to be enriched in the beads contained Ago2, the catalytic component of the RNA induced silencing complex (RISC),^15^ rather than those with IgG in glioma cells (Figure 4D). Seen from Figure 4E, both in U87 and U251 cells, MATN1‐AS1 could be pulled down by Bio‐miR‐200b/c/429‐WT instead of Bio‐miR‐200b/c/429‐MUT or Bio‐NC. In addition, we further demonstrated that MATN1‐AS1 inhibition largely increased the expression of miR‐200b/c/429 (Figure 4F), whereas miR‐200b/c/429 overexpression declined MATN1‐AS1 expression in the two glioma cells (Figure 4G). At length, negative correlations between the expression of MATN1‐AS1 and miR‐200b/c/429 were identified in glioma tissues (Figure 4H). Thus, it is suggested that MATN1‐AS1 can be the sponges of miR‐200b/c/429 in glioma cells.

**Figure 4:** MATN1‐AS1 directly targets miR‐200b/c/429 in glioma cells. A, Three miRNAs which could bind with MATN1‐AS1 are obtained from StarBase database. B, The binding sites between two types of MATN1‐AS1 (wild type and mutant type) and miR‐200b/c/429 were obtained from StarBase database. C, Luciferase reporter assay was conducted to validate the specific binding between MATN1‐AS1 and miR‐200b/c/429 in U87 and U251 cells. D, The complex containing MATN1‐AS1 and miR‐200b/c/429 in U87 and U251 cells was immunoprecipitated by anti‐Ago2 using RIP (RNA immunoprecipitation) assay. E, RNA pull‐down assay was carried out to verify the interactions between MATN1‐AS1 and miR‐200b/c/429. F‐G, The qRT‐PCR results of miR‐200b/c/429 expression in U87 and U251 cells with or without MATN1‐AS1 knockdown (F) and that of MATN1‐AS1 expression in U87 and U251 cells under miR‐200b/c/429 overexpression. H, Spearman's correlation analysis was utilized to evaluate the correlations between the expression of MATN1‐AS1 and miR‐200b/c/429 in glioma tissues. Data are obtained from at least three experiments for mean ± SD. ^*^ *P* < .05, ^**^ *P* < .01 compared with controls. N.S: no significance

The article "MATN1‐AS1 promotes glioma progression by functioning as ceRNA of miR‐200b/c/429 to regulate CHD1 expression" was retracted in 2024. Reasons: errors in the images; plagiarized images; overlap with other authors' work; unreliable results or conclusions.

### 3.6 MATN1‐AS1 regulates CHD1 by sponging miR‐200b/c/429

To find out the possible downstream target of miR‐200b/c/429 which impact glioma, the online tools including TargetScan, PITA, miRanda and RNA22 were employed (Figure S1C). Then, one of the six common target genes of miR‐200b/c/429, the chromodomain helicase DNA‐binding protein 1 (CHD1) which exerts an oncogenic role in ER‐positive breast cancer,^20^ is sorted out due to its important regulatory role in the determination of cell fate.^21^ The binding sites between miR‐200b/c/429 and CHD1 were obtained from online tool TargetScan (http://www.targetscan.org/cgi-bin/targetscan/vert_72/view_gene.cgi?rs=ENST00000284049.3%26taxxml:id=9606%26members=miR-200bc-3p/429%26showcnc=0%26shownc=0%26shownc_nc=%26showncf1=%26showncf2=%26subset=1) (Figure 5A). As displayed in Figure 5B, CHD1 was only remarkably harvested in pellets pulled down by Bio‐miR‐200b/c/429‐WT both in U87 and U251 cells. Subsequently, we observed that the luciferase activity of wild‐type CHD1 was decreased by miR‐200b/c/429 mimics and regained again under MATN1‐AS1 overexpression, whereas that of CHD1‐Mut changes little all the time in U251 cells (Figure 5C). HEK‐293T cells, which had been widely utilized in cell biology research due to their reliable growth and propensity for transfection, were also used here to further validate the interactions among MATN1‐AS1, miR‐200b/c/429 and CHD1. And the luciferase reporter assays conducted in HEK‐293T cells confirm the competitive association between CHD1 and MATN1‐AS1 in binding to miR‐200b/c/429 (Figure 5C). Furthermore, the luciferase activity of CHD1‐WT was increased in U87 and U251 cells only under miR‐200b/c/429 inhibition (Figure 5D). Additionally, pull‐down assay followed by Western blot analysis was performed to determine the interaction between MATN1‐AS1 and CHD1. As a result, no direct interaction between MATN1‐AS1 and CHD1 was analysed (Figure S1D). To explore the relationship between the expression level of MATN1‐AS1, miR‐200b/c/429 and CHD1, we detected their expression in glioma tissues and cell lines, and the downregulation of miR‐200b/c/429 and the upregulation of CHD1 were observed in glioma tissues and cell lines (Figure S2A,B). Then, Spearman's correlation analysis revealed that CHD1 expression was negatively correlated with miR‐200b/c/429 expression but positively related to MATN1‐AS1 level in glioma tissues (Figure 5E). Moreover, we find that both mRNA and protein level of CHD1 in glioma cells were evidently diminished after treating miR‐200b/c/429 mimics while both levels of it were enhanced after miR‐200b/c/429 inhibition (Figure S2C‐G). Meanwhile, both decreased mRNA and protein levels of CHD1 in glioma cells induced by miR/200b/c/429 mimics were recovered by co‐transfection of pcDNA3.1/MATN1‐AS1 (Figure 5F,H). By contrast, the enhanced mRNA and protein levels of CHD1 in glioma cells upon miR‐200b/c/429 inhibition were normalized after silencing MATN1‐AS1 (Figure 5G,I). Hence, our findings declared that MATN1‐AS1 positively modulated CHD1 expression in glioma through sequestering miR‐200b/c/429.

The article "MATN1‐AS1 promotes glioma progression by functioning as ceRNA of miR‐200b/c/429 to regulate CHD1 expression" was retracted in 2024. Reasons: errors in the images; plagiarized images; overlap with other authors' work; unreliable results or conclusions.

**Figure 5:** MATN1‐AS1 regulates CHD1 by sponging miR‐200b/c/429. A, The binding sites between miR‐200b/c/429 and CHD1 were acquired by using bioinformatics analysis. B, RNA pull‐down assay was performed in U87 and U251 cells to confirm the interaction between miR‐200b/c/429 and CHD1. C‐D, Luciferase reporter assay exhibited the interactions among CHD1, miR‐200b/c/429 and in U251 cells and HEK‐293T cells. E, The correlations among CHD1 and MATN1‐AS1 as well as miR‐200b/c/429 in glioma tissues were determined by Spearman's correlation analysis. F‐G, qRT‐PCR was applied to detect changes in the mRNA level of CHD1 in U87 and U251 cells in different groups. H‐I, The changes in CHD1 protein expression levels in U251 cells under different transfections were examined by Western blot analysis. Data are obtained from at least three experiments for mean ± SD. ^*^ *P* < .05, ^**^ *P* < .01 compared with controls. N.S: no significance

### 3.7 CHD1 promotes cell proliferation and inhibits cell apoptosis in glioma cells

Due to the upregulation of CHD1 in glioma tissues and cell lines (Figure S2A,B), we wondered the role of CHD1 in glioma. First of all, the Kaplan‐Meier curve revealed that glioma patients with higher CHD1 expression undergo poorer overall survival than those with lower CHD1 level (Figure 6A). Next, we investigated its effect on the biological behaviours of glioma cells. As displayed in Figure 6B, silencing CHD1 had no influence on MATN1‐AS1 expression but only decreased CHD1 level in both U87 and U251 cells, which verified that CHD1 was the downstream of MATN1‐AS1. Additionally, CHD1 knockdown notably reduced cell viability and colony formation ability in both U87 and U251 cells (Figure 6C,D). Furthermore, the apoptotic rate of two glioma cells was markedly strengthened under CHD1 suppression (Figure 6E). Together, CHD1 silence inhibited cell proliferation but enhances cell apoptosis, namely CHD1‐promoted tumorigenesis in glioma.

The article "MATN1‐AS1 promotes glioma progression by functioning as ceRNA of miR‐200b/c/429 to regulate CHD1 expression" was retracted in 2024. Reasons: errors in the images; plagiarized images; overlap with other authors' work; unreliable results or conclusions.

**Figure 6:** Silencing CHD1 inhibits cell proliferation and induces apoptosis in glioma cells. A, Kaplan‐Meier curve of the correlation between CHD1 expression and overall survival (OS) in patients with glioma. B, qRT‐PCR results of MATN1‐AS1 and CHD1 expression after CHD1 downregulation in U87 and U251 cells. C‐D, Cell proliferative ability of U87 and U251 cells was evaluated by MTT assay and colony formation assay. E, Depletion of CHD1 enhanced cell apoptosis in glioma cells. ^**^ *P* < .01 compared with controls. N.S: no significance

### 3.8 The impact of MATN1‐AS1‐miR‐200b/c/429‐CHD1 axis on glioma cell activities

In order to understand the exact impact of MATN1‐AS1‐miR‐200b/c/429‐CHD1 axis on glioma cell activities, rescue assays were projected and conducted in U251 cells. The results of MTT assay and colony formation assay indicated that the suppressed proliferation in MATN1‐AS1‐downregulated U251 cells was elevated under CHD1 upregulation or miR‐200b/c/429 inhibition (Figure 7A,B). In addition, the increased proportion of U251 cells arrested in G0/G1 phase after MATN1‐AS1 downregulation was reversed upon the co‐transfection of either pcDNA3.1/CHD1 or miR‐200b/c/429 inhibitors (Figure 7C). As displayed in Figure 7D, enhanced cell apoptosis triggered by MATN1‐AS1 silence was rescued after CHD1 overexpression or miR‐200b/c/429 suppression. In the end, the results of Western blot were in accordance with those of flow cytometry analysis (Figure 7E). Taken together, MATN1‐AS1 elicited oncogenic functions in glioma via regulating miR‐200b/c/429‐CHD1 axis.

**Figure 7:** The impacts of MATN1‐AS1‐miR‐200b/c/429‐CHD1 axis on glioma cell activities. A‐B, The proliferation capacity of U251 cells upon different transfections was evaluated by MTT and colony formation assays. C‐D, The changes in cell cycle distribution and apoptosis in indicated U251 cells were tested by flow cytometry analysis. E, Western blot analysis was conducted in transfected U251 cells to further validate above results. Data are obtained from at least three experiments for mean ± SD. ^*^ *P* < .05, ^**^ *P* < .01 compared with controls

The article "MATN1‐AS1 promotes glioma progression by functioning as ceRNA of miR‐200b/c/429 to regulate CHD1 expression" was retracted in 2024. Reasons: errors in the images; plagiarized images; overlap with other authors' work; unreliable results or conclusions.

## 4 DISCUSSION

Recently, increasing evidence has identified that lncRNAs are dysregulated in multiple malignancies.^22^, ^23^, ^24^ Moreover, lncRNAs also modulated biological processes in glioma, such as proliferation, apoptosis and angiogenesis.^25^, ^26^, ^27^, ^28^ MATN1‐AS1 is a newfound lncRNA which locates in 1p35.2 and has been found downregulated in ischaemic stroke.^12^ In this study, we revealed that MATN1‐AS1 was highly expressed in glioma tissues and cell lines, and its upregulation was closely related to poor clinical outcomes. Next, knockdown of MATN1‐AS1 obviously inhibited cell proliferation in vitro and suppresses tumour growth in vivo.

In the past decade, growing evidence has demonstrated that cytoplasmic lncRNAs could function as “RNA sponges” or ceRNAs to bind with miRNAs, and thereby, the regulatory effects of miRNAs on target mRNAs would be hampered.^11^, ^19^ All these reports indicated that there are interactions between miRNAs, lncRNAs and mRNAs in tumours. What's more, it is also elucidated that lncRNAs would influence the progression by sponging miRNAs even in glioma.^10^, ^29^, ^30^, ^31^ Herein, we confirmed the interaction between MATN1‐AS1 and miR‐200b/c/429 as well as their negative correlations in glioma tissues.

CHD1, the chromodomain helicase DNA‐binding protein 1, plays an important role in the determination of chromatin architecture and cell fate.^21^, ^32^ Here, it is screened out as the direct target of miR‐200b/c/429 by using online tools. In addition, CHD1 has been researched to have different effects on different cancers. For example, CHD1 is a tumour suppressor in prostate cancer and oesophageal cancer 33, 34 while it seems to exert as an oncogene in breast cancer.^20^, ^35^ Interestingly, Rodrigues, LU, et al uncover that loss of CHD1 promotes aggressive prostate cancer 36; however, Zhao, D., et al revealed that knockdown of CHD1 inhibits tumour growth of PTEN‐null prostate cancer.^37^ In our study, CHD1 was demonstrated to be an oncogene in glioma and positively regulated by MATN1‐AS1 but negatively regulated by miR‐200b/c/429 in this disease. At last, the rescue assays illustrated that MATN1‐AS1 facilitates glioma progression via miR‐200b/c/429‐CHD1 axis. CHD1 is of considerable importance in DNA repair whose deficiency may eventually cause aberrant expression of multiple oncogenes and tumour suppressors 38; however, the detailed mechanism by which CHD1 regulates genes involved in glioma tumorigenesis needs to be further elucidated in the future.

To sum up, we uncovered that MATN1‐AS1 elicits carcinogenesis through functioning as a ceRNA to regulate CHD1 by sponging miR‐200b/c/429 in glioma for the first time, thereby indicating new targets for glioma treatment. Nevertheless, more researches need to be carried out in the future until applications.

The article "MATN1‐AS1 promotes glioma progression by functioning as ceRNA of miR‐200b/c/429 to regulate CHD1 expression" was retracted in 2024. Reasons: errors in the images; plagiarized images; overlap with other authors' work; unreliable results or conclusions.

## CONFLICTS OF INTEREST

The authors declare that no conflicts of interest are disclosed in this study.

## Data Availability

Research data are not shared.
